# Spatio-Temporal analysis of exports of cultural products and their affecting factors for spatial distribution

This article has been retracted.

**DOI:** 10.1371/journal.pone.0299654

**Published:** 2024-03-14

**Authors:** Xingjia Qie

**Affiliations:** 1 School of Economics, Hebei University, Baoding, Hebei, China; 2 School of Management, Hebei Finance University, Baoding, Hebei, China; University of Education, PAKISTAN

## Abstract

Cultural products constitute a significant portion of global trade, and understanding their export patterns can shed light on economic trends, trade dynamics, and market opportunities. This study conducted the spatio-temporal analysis of exports of cultural products, exploring the relationship between various influencing factors and their impact on the spatial distribution of these exports. Leveraging a diverse dataset encompassing 55 BRI countries for the period of 2005–2022, this research employs advanced spatial analysis techniques, including spatial autocorrelation and spatial regression models, to examine the spatial patterns and determinants of exports if cultural product exports. Moreover, this study delves into the multifaceted determinants affecting the spatial distribution of these exports. The findings of this study reveal significant spatio-temporal variations in the exports of cultural products. Spatial autocorrelation analysis indicates the presence of spatial clustering, suggesting that regions with high cultural product exports tend to be geographically close to each other. The spatial regression models further identify several key factors like economic development, productive capacities, cultural tourism, information development and human capital influence the spatial distribution of these exports. The findings of the study reveal that there is strong spatial relationship for exports of cultural products in BRI countries. The findings of this research contribute valuable insights for policymakers, businesses, and stakeholders regarding a deeper comprehension of the driving forces behind the spatial distribution of these cultural products, facilitating informed decision-making processes to optimize strategies for promoting and sustaining the trade of cultural products in an increasingly interconnected world.

## 1. Introduction

The cultural industry is playing an important role in the global economic development. It generates revenue, creates jobs, and stimulates various sectors of the economy, including tourism, entertainment, media, arts, and crafts [1]. The industry’s growth has a positive impact on GDP and helps diversify the economy beyond traditional sectors. The cultural industry provides employment opportunities for a large number of people, including artists, performers, designers, technicians, marketers, and administrators. It supports both skilled and unskilled workers, contributing to reducing unemployment rates and improving living standards. The cultural heritage and vibrant contemporary cultural scene attract millions of domestic and international tourists [2]. Cultural attractions, festivals, museums, theaters, and cultural events contribute to tourism revenue and foreign exchange earnings. Cultural tourism promotes regional development and stimulates local economies. The cultural industry can contribute to balanced regional development by promoting cultural activities and infrastructure in less-developed areas [3]. It helps bridge the urban-rural divide, reduces regional disparities, and fosters social cohesion by providing cultural opportunities and resources to diverse communities. Recognizing and supporting the cultural industry’s importance can lead to sustainable and inclusive economic development [4].

The United Nations provided a comprehensive delineation of international cultural product and service flow between 1994 and 2003, defining it as the "mode of trade input and output of international cultural products and services." This encompasses not just the import and export of cultural consumer goods but also serves as a crucial vehicle for disseminating ideas, fostering national culture, and amplifying international influence [5]. "Cultural products" encompass a wide array of goods, creations, and expressions that carry cultural significance, reflecting the values, traditions, beliefs, and identities of a particular society or community. These products can be tangible or intangible and cover various domains. Some examples include art and craftwork, literature, music and performing arts, cuisine and food products, fashion and clothing, film and media, religious and spiritual artifacts, language and linguistic artifacts, heritage sites and architecture, traditional knowledge and practices [6]. These cultural products are often deeply rooted in history, tradition, and societal values, serving as tangible or intangible representations of a community’s identity, heritage, and creativity. The export and dissemination of these products contribute to cultural exchange, global diversity, and mutual understanding among different societies and nations [7].

The distinct nature of cultural product trade manifests primarily in the heavily monopolized market of developed nations led by the United States. There’s a lack of unified international standards and tariff constraints, which conceals trade barriers effectively [8]. This uniqueness also lies in the limited openness of sensitive areas within cultural product trade and its seamless integration with other international trade industry products. Understanding this uniqueness holds fundamental value when analyzing the development of cultural product trade [9]. The evolution of cultural product exports has undergone significant transformations over time, influenced by various factors that have shaped trade patterns, technological advancements, and changing consumer behaviors [10]. Centuries ago, cultural products were traded along ancient trade routes such as the Silk Road, connecting civilizations and facilitating the exchange of cultural artifacts. Items like spices, silk, ceramics, and textiles traveled across continents, marking early forms of cultural product exports [11]. During the colonial era, European powers often exploited colonies for resources and cultural goods. This led to the exportation of valuable cultural artifacts, artworks, and materials from colonized regions to the colonizers’ homelands, shaping early global trade in cultural products [12]. The Industrial Revolution transformed production processes, enabling mass production of cultural goods. This led to increased exports of standardized cultural products, such as textiles, art reproductions, and manufactured crafts, to new global markets [13]. The 20th century saw advancements in transportation and communication technology, enabling easier and faster trade in cultural products. This era witnessed the global spread of music, cinema, literature, and fashion, allowing cultural products to reach wider international audiences [14]. Governments began using cultural products as tools for diplomacy and soft power. Cultural exchanges, festivals, and international events aimed at promoting cultural products abroad became common strategies to enhance a country’s image and influence [15]. The rise of the internet and digital technologies revolutionized the export of cultural products. Online platforms enabled the easy dissemination of music, films, literature, and other digital content globally, bypassing traditional distribution channels [16]. Evolving consumer tastes and a growing interest in diverse cultural experiences led to increased demand for authentic and niche cultural products. Consumers seek unique, locally produced items, driving the export of indigenous crafts, traditional cuisines, and ethically sourced goods [17]. Recent trends emphasize sustainability and ethical practices in cultural product exports. Consumers are increasingly interested in products that support fair trade, environmentally friendly production methods, and the preservation of cultural heritage [18]. The COVID-19 pandemic accelerated the shift towards online commerce for cultural products. Lockdowns and restrictions prompted consumers to rely more on e-commerce platforms for purchasing cultural items, influencing trade dynamics [19]. This continuous evolution continues to shape the trade and consumption of cultural goods in the contemporary global marketplace.

The Belt and Road Initiative (BRI) aimed to enhance connectivity and cooperation between countries along its envisioned Silk Road Economic Belt and the 21st Century Maritime Silk Road. The initiative spans various regions, fostering infrastructure development, economic ties, and cultural exchange [20]. The BRI facilitates cultural exchange among participating countries. This exchange extends to the export and import of cultural products such as traditional crafts, artworks, music, films, literature, and fashion, fostering mutual understanding and appreciation of diverse cultures [21]. The BRI promotes cultural tourism, encouraging the export of cultural experiences and heritage sites. It highlights historical landmarks, museums, cultural festivals, and traditional performances, attracting tourists interested in exploring the rich cultural tapestry of BRI countries [22]. Through the BRI, there are initiatives supporting art exhibitions, cultural performances, and exchanges between artists, fostering collaborations and the export of cultural expressions across borders [23]. BRI projects include investments in cultural infrastructure such as museums, theaters, cultural centers, and heritage sites. This development supports the preservation, promotion, and export of cultural products within and beyond the BRI region [24]. The digital realm plays a significant role in exporting cultural products within the BRI region. Digital platforms facilitate the exchange of music, films, literature, and digital artworks, enabling wider access and consumption of cultural expressions [25]. Countries along the BRI often have rich traditions in crafts and artisanal products. The initiative supports the export of traditional crafts, ceramics, textiles, and other handmade goods, promoting cultural heritage and fostering economic opportunities [26]. The BRI’s emphasis on connectivity, infrastructure, and economic cooperation has created opportunities for the export and exchange of cultural products among the diverse countries and regions involved. These cultural exchanges contribute to fostering cultural diversity, mutual appreciation, and economic growth within the BRI framework.

Based on above discussion, there is much importance to study the exports of cultural products and its spatial analysis in the BRI region. Understanding the export dynamics of cultural products in the BRI region facilitates mutual understanding among participating countries. It allows for the appreciation of diverse cultures, traditions, and heritage, fostering stronger cultural ties and mutual respect. Cultural exports represent a significant economic sector. Studying these exports within the BRI helps identify economic opportunities for participating countries. It can lead to the development of strategies to capitalize on cultural strengths, promoting economic growth and job creation. Cultural products serve as tools for soft power and diplomacy. Analyzing their export patterns within the BRI helps understand how countries leverage cultural exports to enhance their global influence, build relationships, and shape perceptions internationally. The BRI involves extensive infrastructure projects that aim to connect participating countries. Studying cultural product exports within this framework allows us to assess how improved infrastructure impacts the movement, accessibility, and trade of cultural goods. Governments can use insights from studying cultural exports to formulate trade policies that support the export of cultural goods. It also informs diplomatic strategies, collaborations, and partnerships between countries, fostering stronger trade relations. Researching cultural exports in the BRI region contributes to academic knowledge across various disciplines, including economics, cultural studies, international relations, and sociology, fostering interdisciplinary insights and collaborations. Moreover, studying the spatial analysis of cultural product exports within the BRI region offers several crucial insights and benefits. Understanding the spatial distribution of exports of cultural product helps to identify regions specializing in certain cultural goods. This knowledge can guide targeted economic development strategies, fostering growth in specific areas and diversifying regional economies. Governments can formulate trade policies tailored to support the export of specific cultural products based on spatial analysis. Policies such as incentives, subsidies, or trade agreements can be designed to boost exports from particular regions. Spatial analysis helps in understanding market trends and consumer behavior in different regions. This knowledge can guide businesses in targeting specific geographical areas for marketing their cultural products effectively.

To explore the spatio-temporal analysis of exports of cultural products and their affecting factors by using the data of 55 BRI economies covering the time span from 2005 to 2022. Then various econometric techniques like Exploratory Spatial Data Analysis and Dynamic Spatial Durbin Panel Model, are applied for empirical analysis. The Dynamic Spatial Durbin Panel Model (DSDPM) offers several advantages in analyzing spatio-temporal relationship. Unlike static models, DSDPM captures dynamic effects by allowing the coefficients to vary over time. This is particularly beneficial for analyzing data with evolving spatial patterns and relationships. DSDPM can handle panel data, which consists of observations over multiple time periods and spatial units. DSDPM also address endogeneity issues by including lagged dependent variables and instrumental variables. It can be used for forecasting future trends and spatial patterns based on historical data and estimated relationships. This can be valuable for decision-makers in anticipating future developments and planning interventions accordingly. Based on empirical estimation, some policies are suggested to promote the trade of cultural products in the BRI region.

## 2. Theoretical foundations

The theoretical foundations underpinning the exports of cultural products encompass various concepts from different disciplines, including economics, sociology, cultural studies, and international trade. Here are some key theoretical frameworks that inform the understanding of exports of cultural product. The cultural economics examines the economic aspects of cultural goods and services. The theory of cultural economics helps understand how supply, demand, pricing, and market structures interact within the cultural sector [27]. It delves into the economic value, consumption patterns, and market behavior related to cultural products. Cultural imperialism theory, rooted in media and cultural studies, explores how dominant cultures exert influence over smaller or less dominant cultures. It considers how powerful nations or cultures shape and control the production, distribution, and consumption of cultural products, impacting their global exports [28]. Cultural globalization theories focus on the spread, exchange, and hybridization of cultural elements across borders. They examine how cultural products transcend national boundaries, influenced by technological advancements, communication networks, and global trade, leading to increased exports of these products [29]. Cultural ecology theory considers the relationship between culture and the environment. In the context of exports of cultural products, it might explore how environmental factors, resources, and sustainability practices influence the production and export of these goods [30]. Commodity chain analysis, often applied in economic geography, studies the entire lifecycle of a commodity, from production to consumption. In the context of cultural products, it examines the complex networks of production, distribution, and marketing involved in exporting these goods [31]. Soft power theory suggests that a country’s cultural attractiveness and influence can be more persuasive than military or economic power. Cultural diplomacy utilizes cultural products as tools for international relations, impacting their export strategies [32]. Cultural protectionism theory concerns policies aimed at safeguarding a nation’s cultural heritage and industries. It involves implementing regulations, subsidies, or quotas to protect domestic cultural products from being overwhelmed by foreign imports. Theoretical frameworks in psychology and marketing help understand consumer preferences, attitudes, and behavior regarding cultural products. These theories explore how perceptions of authenticity, identity, and cultural significance influence purchasing decisions [33]. Network theory focuses on the interconnectedness of actors and institutions in the production and distribution of cultural products. It examines how networks of producers, distributors, consumers, and policymakers influence the export of cultural goods [34]. Classical economic theories like comparative advantage explain how countries specialize in producing goods and services where they have an advantage. Applied to cultural products, this theory can highlight why certain regions become primary exporters due to their cultural expertise or resources [35]. These theoretical foundations provide lenses through which scholars and policymakers analyze, interpret, and navigate the complexities surrounding the export dynamics of cultural products within the global marketplace.

## 3. Methodology

### 3.1. Exploratory Spatial Data Analysis (ESDA)

ESDA is a methodology used to analyze and understand spatial data patterns, relationships, and structures. It focuses on exploring spatial datasets to uncover potential spatial trends or clusters. ESDA examines spatial autocorrelation, which assesses the similarity of values between neighboring locations. It helps identify if similar values tend to cluster together or if there’s spatial randomness. This analysis is crucial for understanding whether spatial patterns exist and if there’s any dependency between neighboring observations. Analyzing spatial relationships involves assessing how the proximity or distance between locations affects their attributes. Understanding these relationships can reveal insights into phenomena like spatial dependence, clustering, or spatial outliers, providing valuable information for decision-making and policy planning. ESDA often involves hotspot analysis to identify statistically significant clusters of high or low values in a dataset.

Spatial dependence models offer several advantages in analyzing spatial data. Spatial dependence models explicitly account for spatial relationships among observations, considering how proximity or distance between locations influences the variable of interest [36]. This enables a more accurate representation of the underlying spatial structure. By incorporating spatial dependencies, these models can provide more accurate predictions or estimations, especially when the variable being analyzed exhibits spatial clustering or autocorrelation. This improves the model’s predictive power compared to traditional non-spatial models. Spatial dependence models can handle spatial heterogeneity, acknowledging that observations in different locations might have unique characteristics or relationships [37]. This flexibility helps accommodate variations across spatial units. These models are effective in identifying clusters, hotspots, or spatial outliers within a dataset. They can pinpoint areas with unusually high or low values, aiding in the identification of spatial patterns and anomalies. Spatial dependence models facilitate better inference by addressing spatial autocorrelation or dependency in the data. This helps in producing more reliable statistical estimates and inferences, avoiding biased parameter estimates due to spatial effects [38]. For applications in urban planning, environmental management, or public health, understanding spatial relationships is crucial. Spatial dependence models assist in formulating policies and interventions tailored to specific spatial patterns and clusters. In regression modeling, spatial dependence models can address spatially correlated errors, accounting for the interdependence among residuals that might arise due to unobserved spatial factors [39]. Moran’s I values is used to measure the intensity of spatial dependence.

Global spatial autocorrelation refers to the assessment of spatial patterns across an entire geographic area or dataset. It evaluates the degree of similarity or dissimilarity of attribute values among all locations in a spatial dataset [40]. This analysis provides an overall understanding of the spatial dependence within the entire dataset rather than focusing on specific regions or clusters. The primary goal is to determine if there’s a systematic spatial pattern across the entire study area, whether similar values are clustered together, dispersed, or randomly distributed [41]. Common measure used to assess global spatial autocorrelation includes Moran’s I. These statistics evaluate the spatial relationships among all observations and provide a single value indicating the strength and direction of spatial association within the entire dataset. A high positive Moran’s I value, for instance, suggests that similar values tend to be near each other, indicating clustering or spatial concentration. Conversely, a negative Moran’s I value might suggest a dispersed or random pattern. The “GM’s I” test is specified as:

$$I=\frac{n\sum_{i=1}^{n}\sum_{j=1}^{n}W_{ij}(x_{i}-\bar{x})(x_{j}-\bar{x})}{\sum_{i=1}^{n}\sum_{j=1}^{n}W_{ij}\sum_{i=1}^{n}{\left(x_{i}-\bar{x}\right)}^{2}}$$

In above equation, n is number of countries, x_i_ and x_j_ represent culture products in i and j countries, Wij is spatial weight matrix (SWM). Rook contiguity, k-nearest neighbors, and queen contiguity are few algorithms used to judge the adjacent relationships. The rook contiguity is used for construction of row standardized SWM. The value of GM’s I near to 1 reveals the strong positive spatial correlation while value closer to -1 highlights the strong negative spatial correlation.

The “spatial autocorrelation model” (SAC), “spatial error model” (SEM), and “spatial autoregressive model” (SAR) are different categories of spatial econometric model.

The Dynamic Spatial Durbin Panel Model (DSDPM) is a sophisticated econometric framework used to analyze panel data where both spatial and temporal dependencies exist. This model is an extension of the Spatial Durbin Model (SDM) and incorporates time-varying factors, allowing for the examination of spatial interactions and temporal dynamics simultaneously. DSDPM works with panel datasets, which contain observations on multiple entities over multiple time periods. It considers both cross-sectional and time-series dimensions, capturing spatial interactions and temporal changes within the data. Similar to the Spatial Durbin Model, DSDPM accounts for spatial interdependence among different spatial units, acknowledging that the values of a variable in one location can be influenced by the values in neighboring locations. DSDPM extends the SDM by incorporating time-varying effects, allowing for the investigation of how both spatial interactions and temporal changes affect the variable of interest over time. It addresses endogeneity issues by including lagged values of the dependent variable and spatially lagged values of the explanatory variables, accounting for the potential feedback effects and addressing simultaneity concerns. The model typically includes spatial lag terms, temporal lag terms, and spatiotemporal interaction terms, providing a comprehensive framework to capture the complex interplay between space and time. Estimation of the DSDPM involves accounting for spatial autocorrelation, heterogeneity, and potentially correlated errors across space and time, requiring advanced statistical techniques for parameter estimation. The DSDP Model offers a powerful framework to analyze the complex interdependencies between space and time in panel data settings, providing valuable insights into how spatial interactions and temporal dynamics jointly influence outcomes over time. Spatial Durbin model (SDM) includes the spatial lag terms of dependent and independent variables [33], and the formula is as follows:

$$y_{it}=\partial_{0}+\partial_{1}y_{i,t-1}+\eta \sum_{j=1}^{n}W_{ij}y_{j,t-1}+\rho \sum_{j=1}^{n}W_{ij}y_{jt}+\partial_{2}X_{it}+\partial_{3}\sum_{j=1}^{n}W_{ij}X_{jt}+\mu_{i}+\xi_{t}+\varepsilon_{it}$$

In above equation, y_it_ denotes the explained variable, W_ij_ is SWM, α1 shows time lag coefficient. ρ is spatial autoregressive coefficient, η is spatio-temporal lag coefficient, X is independent variable, μ_i_ is regional fixed effect, ξ_t_ is time fixed effect, and ε_it_ is random error term.

### 3.2. Data

The annual panel data of 55 BRI economies is used covering the time span of 2005–2022. The sample is selected on the basis of data availability while data sources and measurement of variables are mentioned in the following Table 1.

**Table 1:** Variables.

Variable	Symbol	Measurement	Sources
Export of Cultural Products	ECP	Percentage of Total exports of Services	UNCTAD
Economic Development	ECD	Per capita GDP	WDI
Globalization	GLZ	KOF Index	KOF Swiss Economic Institute
Information Development	IND	Total volume of Post and Telecommunications Business	WDI
Productive Capacities	PRC	Index	UNCTAD
Cultural Tourism	CLT	Expenditures on Cultural Tourism as percentage of GDP	WDI
Human Capital	HCP	Per capita wages of employees	WDI

### 3.3. Empirical findings

Table 2 shows the values of GM’s I index.

**Table 2:** GM’s I index for exports of cultural products.

**Years**	**2005**	**2006**	**2007**	**2008**	**2009**	**2010**	**2011**	**2012**	**2013**
GM’s I	0.349	0.322	0.369	0.408	0.431	0.277	0.388	0.371	0.422
p value	0.000	0.001	0.002	0.002	0.000	0.003	0.001	0.002	0.001
z value	4.573	5.147	5.422	5.472	5.259	4.585	4.754	5.138	6.288
**Years**	**2014**	**2015**	**2016**	**2017**	**2018**	**2019**	**2020**	**2021**	**2022**
GM’s I	0.482	0.438	0.469	0.471	0.396	0.325	0.401	0.433	0.442
p value	0.000	0.002	0.002	0.003	0.002	0.001	0.000	0.001	0.002
z value	5.556	5.473	5.537	6.142	5.426	6.270	5.481	4.534	5.471

The Z values show the spatial dependence of exports of cultural products. So spatial model is superior as compared with classic model.

### 3.4. Influencing factors of exports of cultural products

Prior to estimate the model, stationarity test is conducted to prevent spurious regression. The unit root tests including Levin-Lin-Chu (LLC) and ADF-Fisher, indicated that at a 1% significance level, all variables except per capita GDP and information development rejected the null hypothesis at level. Then first-order unit root test was necessary for all variables. The outcomes revealed that all variables rejected the null hypothesis at a 1% significance level. Subsequently, co-integration tests were performed. Both Kao and Pedroni tests rejected the null hypothesis at a 1% significance level, indicating a long-term stable relationship among variables. Moreover, the Hausman test is employed and P-statistic value of 0.000 suggests that the spatial econometric model with fixed-effects better elucidates the relationship between the dependent variable and its influencing factors. The Wald (SAE) and LR (SEM) statistics, 54.42 and 31.75 respectively, rejected both the hypotheses of θ = 0 and θ = -βρ, underscoring the high goodness of fit of the SDM model.

The regression outcomes, shown in Table 3, affirm that SDM is an excellent model for comprehending the impacts of exogenous variables on the dependent variable, evident from its highest adjusted R2 value and lowest HQ, SC, and AIC values. To validate the empirical findings, four spatial models were employed using different spatial weight matrices, including ’Queen based contiguity weight matrix,’ ’K nearest contiguity weights matrix,’ and ’double rook contiguity weight matrix.’ The LR test and goodness of fitness consistently support the superiority of the SDM over other spatial models. The results of the chosen spatial weight matrix are presented in Table 3.

**Table 3:** Spatial models.

Variables	Model 1	Model 2	Model 3	Model 4
ECD	0.468*(0.019)	0.378*(0.011)	0.417* (0.019)	0.467*(0.010)
GLZ	0.049 (0.052)	0.043 (0.072)	0.051 (0.052)	0.087***(0.042)
IND	0.212**(0.025)	0.243***(0.019)	0.222**(0.0211)	0.213*(0.0198)
PRC	0.337**(0.086)	0.044**(0.088)	0.325**(0.099)	0.295**(0.092)
CLT	0.025* (0.004)	0.028*(0.003)	0.020* (0.003)	0.029* (0.005)
HCP	0.042*(0.004)	0.051*(0.003)	0.044*(0.004)	0.049*(0.002)
Constant	1.843**(0.227)	3.753**(0.322)	4.352**(0.173)	5.864**(0.732)
Spatial Effect				
Α		0.047(0.042)	0.065(0.036)	0.274(0.072)
Φ	0.562**(0.056)		0.375**(0.062)	
W*ECD				-0.632*(0.041)
W*GLZ				-0.075(0.887)
W*IND				-0.836***(0.049)
W*PRC				-0.756*(0.034)
W*CLT				-0.026**(0.023)
W*HCP				0.036**(0.213)
Model Fitness				
F-statistics	485.32**	563.52*	475.42*	526.43*
p-value (F-statistics)	0.002	0.004	0.003	0.002
R^2^	0.932	0.929	0.921	0.972
Adjusted R^2^	0.911	0.914	0.901	0.952
HQ	0.434	0.316	0.327	0.273
SC	0.475	0.446	0.507	0.221
AIC	0.403	0.315	0.442	0.254

Note

*, **, and *** show significance level at 1%, 5% and 10% respectively.

The empirical findings show that lagged dependent variable has a positive relationship. The estimated value conveys that one-unit increase in exports of cultural products of neighboring countries increases the exports of cultural products in own state by 0.274 unit.

Several robustness tests are conducted to evaluate the credibility and consistency of model. Lagrange Multiplier Test detects potential omitted variable bias within the model by assessing the null hypothesis of no spatial dependence. Rejecting this hypothesis suggests the presence of omitted variable bias, indicating the model’s inadequacy in accounting for spatial relationships. The Variance Inflation Factor (VIF) test identifies multicollinearity among independent variables. High VIF values signal a high correlation between these variables, which can complicate the estimation of model coefficients. The Cross-Validation test make partitions of the data into training and testing sets to evaluate the model’s predictive performance. If the model effectively predicts values in the testing set, it signifies the model’s robustness and reliability in its predictive capacity.

## 4. Discussion

This paper explored the various aspects of exports of cultural products of 55 BRI countries from 2005 to 2022. We evaluated the spatio-temporal characteristics of culture products and also analyzed the influencing factors of exports of cultural products. There is strong spatial impact of exports of cultural products in the region. The findings of the study reveal that economic development positively influences the exports of cultural products. Economic growth generally leads to higher disposable incomes. As countries develop economically, consumers often have more purchasing power, leading to increased demand for cultural products. This elevated demand fuels the export of cultural items like music, films, literature, and art to cater to international markets [42]. Countries experiencing economic prosperity tend to invest in their creative sectors, leading to the production of high-quality cultural products. Strong domestic production lays the foundation for competitive exports, as these products gain international appeal. Economically developed countries often have robust trade networks and better access to global markets [43]. This facilitates the export of their cultural products, enabling them to penetrate various international markets effectively. Globalization allows cultural exports to reach diverse audiences worldwide. Economic progress often translates into investments in cultural infrastructure, such as theaters, museums, studios, and publishing houses [44]. These investments contribute to the production, promotion, and export of cultural goods by providing necessary platforms and resources for artists and creators. Economic development strengthens a country’s ability to engage in cultural diplomacy. Culturally rich nations utilize their exports of music, cinema, literature, and other cultural products to exert soft power, shaping international perceptions and fostering relationships with other nations [9, 45]. Economic growth allows governments to allocate resources and implement supportive policies for the cultural sector. Subsidies, grants, and incentives provided to artists and cultural industries encourage the creation and export of cultural products [46].

Economic development shapes the cultural exports by influencing production capacities, market dynamics, and policies. This, in turn, leads to spatial implications, with certain regions becoming hubs for cultural production and export, while others may face challenges related to regional disparities or the preservation of cultural identity [33, 47]. Certain regions become specialized in specific cultural domains due to economic development and historical factors. Developed regions often have superior infrastructure, such as transport networks and digital connectivity, facilitating the export and dissemination of cultural products more efficiently [24, 48]. Economic development might exacerbate regional disparities. Stronger economies may dominate cultural exports, leading to unequal distribution of cultural influence and economic benefits across regions within a country. In some cases, regions experiencing economic growth may prioritize the preservation and export of their unique cultural identity, promoting localized cultural exports that distinguish them in the global market [16, 49]. Economic development can foster tourism in culturally rich regions, leading to increased exposure and demand for local cultural products, subsequently influencing export patterns from these areas. Regions with stronger economies often have better government support and policies for cultural industries, creating conducive environments for the creation and export of cultural goods [21, 50].

The findings of the study highlight that globalization has significant positive impact on export of cultural products, influencing both the nature of cultural exports and their spatial distribution. Globalization opens up international markets, providing opportunities for cultural products to reach a broader audience [51]. This leads to increased export potential for various cultural items such as music, films, literature, and art across borders. It can lead to a dual effect. On one hand, it fosters cultural homogenization by promoting more commercially viable, standardized products that appeal to global audiences [14, 52]. On the other, it encourages the export of diverse cultural products, allowing for the representation of various cultural identities and expressions. Globalization is intertwined with technological advancements, facilitating the distribution and accessibility of cultural products through digital platforms, streaming services, and social media, creating new channels for export. Nations use cultural exports as a means of projecting soft power globally [22, 53]. Culturally rich countries utilize their exports of music, cinema, literature, and art to influence global perceptions and enhance their international influence. Globalization fosters cultural exchange and fusion. Cultural products often reflect hybrid identities, blending elements from various cultures, which can enhance their export appeal to diverse audiences [54].

Information development, particularly advancements in technology and communication, significantly increase the export of cultural products. Information development fosters improved digital connectivity, enabling easier access to global markets for cultural products [55]. Advancements in information technology provide platforms like streaming services, social media, and e-commerce, offering new channels for cultural product distribution and reaching global audiences. Improved information infrastructure encourages cross-border collaboration among artists, filmmakers, writers, and creators [14, 56]. This collaboration enhances cultural products and expands their export potential. Information technologies facilitate more sophisticated marketing strategies, enabling the countries to better promote their cultural exports globally, increasing visibility and demand for their products. Technological advancements encourage the creation of unique and competitive cultural products suitable for export. Strengthened information development contributes to economic growth, fostering a conducive environment for cultural industries [11, 57]. This economic progress supports increased exports of cultural goods.

Information development influences the spatial impact by enhancing connectivity along the BRI corridors, facilitating the movement of cultural products across regions and trade routes. Information development within BRI countries significantly impacts the export of cultural products by improving digital connectivity, enhancing marketing capabilities, fostering innovation, and preserving cultural heritage [58]. These advancements have spatial implications, influencing trade routes, creative clusters, and the economic dynamics of regions along the BRI corridors.

Productive capacities have also positive impact on exports of cultural products. Strong productive capacities enable the countries to produce a diverse range of high-quality cultural products because it allows to adopt modern production techniques and create culturally appealing, technologically advanced products suitable for global export [18, 59]. It contributes to the development of creative industries. Adequate resources, skilled labor, and technological infrastructure foster a conducive environment for cultural production. Strong productive capacities often correspond to economic stability, attracting investments in the cultural sector. This leads to increased production, innovation, and competitiveness in exporting cultural goods [26, 60]. Enhanced productive capacities encourage innovation and adaptability within the creative sectors. This enables the creation of culturally relevant and adaptable products that cater to diverse global audiences.

Cultural tourism significantly impacts the export of cultural products, influencing both the demand for and promotion of cultural goods. Cultural tourism stimulates interest in the unique heritage, traditions, and artistic expressions. Visitors seek authentic cultural experiences, creating demand for locally produced cultural products such as handicrafts, traditional arts, music, and literature [17, 61]. Tourists become potential consumers of cultural products, seeking souvenirs and memorabilia that represent the visited destination’s cultural identity. This exposure expands the market for cultural goods, often leading to increased exports. Cultural tourism serves as a promotional tool for cultural exports. Visiting tourists become ambassadors, purchasing and showcasing cultural products in their home countries, thereby indirectly promoting exports [29, 62]. It fosters the preservation and commercialization of cultural heritage. Local artisans and craftsmen produce traditional items for sale to tourists, leading to a commercial market for cultural products. In response to tourist demands, BRI countries often diversify their cultural offerings. This could lead to the creation of new products or adaptations of traditional ones, catering to the preferences of diverse tourist demographics [31, 63]. In summary, cultural tourism acts as a catalyst for the export of cultural products in BRI countries. It generates demand, provides exposure, promotes cultural exports, and influences the spatial dynamics by fostering cultural markets, artistic clusters, and economic zones catering to tourist interests.

Human capital plays a pivotal role in exports of cultural products in BRI countries. Skilled human capital, including artists, writers, designers, and technicians, forms the backbone of cultural production [19, 44]. Countries with a well-educated and skilled workforce are better equipped to produce high-quality cultural products. Human capital drives innovation in creative industries within BRI countries. Well-trained professionals are instrumental in adapting to technological advancements, creating innovative cultural products suitable for global export. Educated and culturally aware individuals contribute to the preservation and revitalization of traditional arts and heritage [13, 21]. This authenticity adds value to cultural products, making them more attractive for export. Human capital with marketing, promotion, and business skills is crucial in effectively promoting and exporting cultural products. Proficient professionals can navigate global markets, enhancing the visibility and reach of cultural exports. Human capital possessing multilingual and cross-cultural skills can effectively communicate and tailor cultural products to diverse global audiences, facilitating export and market penetration [12, 37]. The presence of skilled professionals, educational institutions, creative hubs, and talent clusters impacts the spatial dynamics by fostering creative centers and networks crucial for the export of cultural goods.

## 5. Conclusion

This study is an effort to explore the spatio-temporal analysis of exports of cultural products in 55 BRI countries covering the time span from 2005–2022. The analysis offers valuable insights for cultural product exports and their influencing factors, elucidating their impact on spatial distribution. As evidenced by this comprehensive exploration, the export of cultural products is a multifaceted phenomenon shaped by a myriad of interrelated elements, encompassing economic, social, and technological dimensions across various regions and temporal frames. Through this analysis, it becomes evident that the export of cultural products transcends mere economic transactions; it embodies the essence of identity, heritage, and creativity within nations. The spatial distribution of these exports is a testament to the intricate interplay between regional specializations, human capital, technological advancements, and global market dynamics. Moreover, the spatio-temporal patterns unveiled herein underscore the significance of regional clusters, urban centers, and specialized hubs in fostering the production, innovation, and export of cultural goods. These spatial dynamics not only reflect the richness and diversity of cultural expressions but also highlight the economic potential embedded within creative industries across different geographies. Nevertheless, the findings also illuminate certain challenges and disparities, underscoring the need for strategic interventions. Bridging the gap in human capital, leveraging technological advancements, and fostering cross-border collaborations are imperative for achieving a more equitable and sustainable distribution of cultural exports within and between regions. As we navigate an increasingly interconnected global landscape, understanding the spatio-temporal nuances of cultural product exports is pivotal. This analysis serves as a foundation for policymakers, stakeholders, and industry leaders to formulate informed strategies, promoting cultural exchange, economic growth, and the preservation of cultural heritage while fostering a more balanced and inclusive spatial distribution of cultural exports. Ultimately, it is through a holistic and collaborative approach that the true potential of cultural exports can be harnessed to enrich societies and economies on a global scale.

### 5.1. Practical implications

Governments can utilize the findings to tailor trade policies specifically targeting the export of cultural products. This could involve providing incentives, subsidies, or support to industries involved in the production of these cultural goods. Understanding the spatial distribution of exports can aid in identifying regions that specialize in certain cultural products. This knowledge can inform economic development strategies, encouraging the growth of these industries in specific areas, thereby boosting regional economies. Businesses involved in the production and export of cultural products can benefit from insights into the temporal patterns and factors affecting export. This information can guide their market strategies, such as determining the best times to export or identifying factors that impact market demand. Insights from the analysis help in preserving cultural heritage and traditions. By understanding which cultural products are being exported and from which regions, efforts can be made to safeguard and promote these unique cultural expressions. Governments and investors can use this analysis to determine where to allocate resources and infrastructure to support the production and export of cultural goods. For instance, investing in transportation or logistics in regions identified as significant exporters could improve efficiency. Understanding the dynamics of cultural exports can also impact international relations. It can foster collaborations and partnerships between countries with shared interests in certain cultural products, leading to cultural exchange programs or trade agreements. Cultural exports often tie into a country’s tourism appeal. Knowledge about the export patterns and factors affecting cultural products can be utilized in tourism campaigns to attract visitors interested in experiencing or purchasing these unique cultural items. Academia and researchers can benefit from the analysis to delve deeper into the socio-economic factors influencing the production and export of cultural goods. This could lead to further studies, creating a cycle of continuous learning and improvement in understanding these dynamics.

### 5.2. Limitations

The analysis heavily relies on available data. Limitations in data collection, inconsistencies, or inaccuracies in data can undermine the reliability and generalizability of the findings. Cultural trends and trade patterns can evolve rapidly. The study’s reliance on a specific time frame might not capture the dynamic nature of cultural exports, potentially making its conclusions outdated or less relevant over time. Certain cultural products might have ethical or sensitive aspects related to their production, export, or consumption. The study may not delve into these nuanced ethical dimensions adequately. Shifts in trade policies, geopolitical landscapes, or cultural dynamics could significantly impact cultural exports. The study’s findings might become obsolete or less applicable due to changes in the external environment. The future study might thoroughly consider human behavior, consumer preferences, or individual choices that influence the demand and export of cultural products.

## References

[1] RichardsG. Cultural attractions and European tourism. 1st ed. Cambridge: CABI Publishing; 2001.

[2] JohnU. The tourist gaze. Leisure and travel in contemporary societies. 1st ed. London: Sage Publications; 1990.

[3] McIntoshRW, GoeldnerCR. Tourism: principles, practices, philosophies. Shanghai Shanghai Cultural Press; 1985.

[4] XuJ. Tourism culture and cultural tourism: Some problems in theory and practice. Tourism Tribune. 2005; 20(4):67–72.

[5] RichardsG. Culture and tourism: natural partners or reluctant bedfellows? A perspective paper. Tourism Review. 2020; 75(1):232–234.

[6] CorteseF, D’AmbrosioI, PetraccaM. A Possible Synergy between Culture and Religion for the Sustainability of Tourism of Pompeii. Sustainability. 2019; 11(8):2231.

[7] AlbertiFG, GiustiJD. Cultural heritage, tourism and regional competitiveness: The Motor Valley cluster. City, Culture and Society. 2012; 3(4):261–273.

[8] RichardsG. Creativity and tourism: The State of the Art. Annals of Tourism Research. 2011; 38 (4):1225–1253.

[9] WuJ, SongZ. Study on the development of movie-induced tourism from the perspective of industrial merging. Tourism Tribune. 2011; 26(6):29–35.

[10] RichardsG. Creativity and tourism in the city. Current Issues in Tourism. 2014; 17(2):119–144.

[11] QuC, TimothyDJ, ZhangC. Does tourism erode or prosper culture? Evidence from the Tibetan ethnic area of Sichuan Province, China. Journal of Tourism and Cultural Change. 2019; 17(4):526–543.

[12] MaX, WangR, DaiM, OuY. The influence of culture on the sustainable livelihoods of households in rural tourism destinations. Journal of Sustainable Tourism. 2021; 29(8):1235–1252.

[13] SuZ, AaronJR, McDowellWC, LuD. Sustainable synergies between the cultural and tourism industries: An efficiency evaluation perspective. Sustainability. 2019; 11(23):6607.

[14] SeoJH, KimB. The “Hallyu” phenomenon: Utilizing tourism destination as product placement in K-POP culture. Tourism Economics. 2020; 26(4):719–728.

[15] WhangH, YongS, KoE. Pop culture, destination images, and visit intentions: Theory and research on travel motivations of Chinese and Russian tourists. Journal of Business Research. 2016; 69(2):631–641.

[16] LarsonM, LundbergC, LexhagenM. Thirsting for vampire tourism: Developing pop culture destinations. Journal of Destination Marketing & Management. 2013; 2(2):74–84.

[17] WuL, liangH, YuH, HuoR. Spatial differentiation and driving factors of the integrated development of culture and tourism in China. Economic Geography. 2021; 41(2):214–221.

[18] KongY. The path selection of the integration development of tourism industry and cultural industry: Taking Hebei Province as an example. Social Science Forum. 2016;(10):240–244.

[19] MaY, TongY. From the region to domain: Re-understanding the relationship between culture and tourism. Tourism Tribune. 2019; 34(4):7–9.

[20] ZhangC, ZhuM. The integration of culture and tourism: Multi-understandings, various challenges and approaches. Tourism Tribune. 2020; 35(3):62–71.

[21] BaoH, WangS. Coupling analysis of cultural industry and tourism industry. Industrial Technology and Economy. 2010; 29(08):74–78.

[22] LiS, DuS. An Empirical Study on the Coupling Coordination Relationship between Cultural Tourism Industry Competitiveness and Tourism Flow. Sustainability. 2021; 13(10):5525.

[23] FanT, XueD. Spatial correlation of cultural industry and tourism industry in Shaanxi Province, China: LISA analysis based on coordination model. Asia Pacific Journal of Tourism Research. 2020; 25 (9):967–980.

[24] WengG, LiL. The coupling coordination degree and spatial correlation analysis on integrational development of tourism industry and cultural industry in China. Economic Geography. 2016; 36(1):178–185.

[25] BaD. 40 years of reform and opening-up: The value and trend of the integration of chinese cultural tourism. Social Sciences in Gansu. 2018;(5):10–20.

[26] ZhangS. The internal mechanism, basic model and industrial development logic of the in-depth integration of cultural industries and tourism. Journal of China University of Petroleum (Edition of Social Sciences). 2019; 35(5):94–99.

[27] LiebowitzSJ, MargolisSE. The fable of the keys. Journal of Law and Economics. 1990; 31(1):1–25.

[28] HuangR, XuJ. Efficiency lock-in and efficiency change of industrial development: based on the integration of "cultural tourism" industry. Jianghan Tribune. 2020;(8):37–45.

[29] SextonTR, SilkmanRH, HoganAJ. Data envelopment analysis: Critique and extensions. New Directions for Program Evaluation. 1986; (32):73–105.

[30] DoyleJ, GreenR. Efficiency and cross-efficiency in DEA: Derivations, meanings and uses. Journal of the Operational Research Society. 1994; 45(5):567–578.

[31] GatrellAC. Autocorrelation in spaces. Environment and Planning A: Economy and Space. 1979; 11 (5):507–516.

[32] AnselinL. Local indicators of spatial association—LISA. Geographical Analysis. 1995; 27(2):93–115.

[33] ElhorstJP. Dynamic spatial panels: models, methods, and inferences. Journal of Geographical Systems. 2012; 14(1):5–28.

[34] DengY, YouD, WangJ. Research on the nonlinear mechanism underlying the effect of tax competition on green technology innovation—An analysis based on the dynamic spatial Durbin model and the threshold panel model. Resources Policy. 2022; 76:102545.

[35] XieK. Uncertainty convergence and optimization of system: on the management science of non-system. Journal of Sun Yatsen University (Social Science Edition). 2005; 45(2):90–96.

[36] ZhangY, CuiQ. The integration evaluation between industrialization and informatization in China. Science Research Management. 2013; 34(4):43–49.

[37] YanS, MiaoJ. Study on the integration efficiency between high-tech industry and traditional industry of urban agglomeration in the middle reaches of Yangtze River. Science and Technology Management Research. 2017;(12):66–72.

[38] CaoF, HuangZ, WuJ, XuM. The space-time pattern evolution and its driving mechanism of urban tourism development efficiency: A case study of Pan-Yangtze River Delta. Georaphical Research. 2012; 31 (8):1431–1444.

[39] QinW, ZhangY, LiS. Study on the spatio-temporal evolution of coastal city tourism of China. Geographical Research. 2014; 33(10):1956–1965.

[40] WangW, GuJ. Evolution of Time and Space Efficiency of Cultural Industry in the Yangtze River Economic Belt. Nanjing Journal of Social Sciences. 2021;(6):169–178.

[41] ZhangJ, HouZ, LiuP, HeJ, ZhuoX. The goals and strategic path of high-quality development. Management World. 2019; 35(7):1–7.

[42] ZhangT, WuJ. Spatial Network Structure and Influence Mechanism of Green Development Efficiency of Chinese Cultural Industry. Scientia Geographica Sinica. 2021; 41(4):580–597.

[43] WangR, XiaB, DongSC, LiY, LiZH, BaDX, et al. Research on the Spatial Differentiation and Driving Forces of Eco-Efficiency of Regional Tourism in China. Sustainability. 2021; 13(1):280.

[44] HalkosGE, TzeremesNG. National culture and eco-efficiency: an application of conditional partial nonparametric frontiers. Environmental Economics and Policy Studies. 2013; 15(4):423–441.

[45] LiJ, LiaoJ. Research on influencing factors of the development of cultural and creative industries based on grey factor analysis. Computer Science and Information Systems. 2021; 18(4):1253–1269.

[46] CaoF, HuangZ, JinC, XuM. Influence of Chinese economic fluctuations on tourism efficiency in national scenic areas. Tourism Economics. 2016; 22(5):884–907.

[47] LiuZ, LuC, MaoJ, SunD, LiH, LuC. Spatial–Temporal Heterogeneity and the Related Influencing Factors of Tourism Efficiency in China. Sustainability. 2021; 13(11):5825.

[48] GetisA, OrdJK. The analysis of spatial association by use of distance statistics. Geographical Analysis. 1992; 24(3):189–206.

[49] BoxJF. Guinness, Gosset, Fisher, and Small Samples. Statistical Science. 1987; 2(1):45–52.

[50] LeSageJ, PaceRK. Introduction to spatial econometrics. 1st ed. New York: Chapman and Hall/CRC; 2009.

[51] MoY.; MadniG.R. Pollution halo impact in context of productive capacities, energy poverty, urbanization, and institutional quality. PLoS ONE. 2023, 18(12), e0295447. doi: 10.1371/journal.pone.0295447 38060540 PMC10703264

[52] ChenQ.; MadniG.R. Greening the BRI countries through economic and political reforms. PLoS ONE. 2023, 18(11), e0294967. doi: 10.1371/journal.pone.0294967 38015953 PMC10684069

[53] ChenQ.; MadniG.R.; ShahzadA.A. The usage of spatial econometric approach to explore the determinants of ecological footprint in BRI countries. PLoS ONE. 2023, 18(10), e0288683. doi: 10.1371/journal.pone.0288683 37906557 PMC10617693

[54] MadniG.R. Meditation for role of productive capacities and green investment on ecological footprint in BRI countries. Environmental Science and Pollution Research. 2023, 30(28), 72308–72318. doi: 10.1007/s11356-023-27478-0 37170048

[55] MellanderC.; FloridaR. The rise of skills: Human capital, the creative class, and regional development. In Handbook of Regional Science; FischerM., NijkampP., Eds.; Springer: Berlín, Germany, 2018.

[56] AnderssonÅ.E.; AnderssonD.E.; DaghbashyanZ.; HårsmanB. Location and spatial clustering of artists. Reg. Sci. Urban. Econ. 2014, 47, 128–137.

[57] ŽenkaJ.; SlachO.; IvanI. Spatial patterns of knowledge-intensive business services in cities of various sizes, morphologies and economies. Sustainability. 2020, 12, 1845.

[58] LazzerettiL.; CaponeF.; BoixR. Reasons for clustering of creative industries in Italy and Spain. Eur. Plan. Stud. 2012. 20, 1243–1262.

[59] HongJ.; YuW.; GuoX.; ZhaoD. Creative industries agglomeration, regional innovation and productivity growth in China. Chin. Geogr. Sci. 2014. 24, 258–268.

[60] Cliff, A.; Ord, D. Spatial Processes: Models and Applications; Pion: London, UK, 1981.

[61] GarcíaM.I.; FernándezY.; ZofíoJ.L. The economic dimension of the culture and leisure industry in Spain: National, sectoral and regional analysis. J. Cult. Econ. 2003. 27, 9–30.

[62] BoalI.; HerreroL.C. Where are the artists? Analysing economies of agglomeration in Castile and León, Spain. Pap. Reg. Sci. 2018. 97, 995–1016.

[63] XuB.C.; PanJ.H. Spatial distribution characteristics of the intangible cultural heritage in China. Econ Geogr. 2018, 38(05), 188–196.

